The article "Hybrid Optimized GRU-ECNN Models for Gait Recognition with Wearable IOT Devices" was retracted in 2023. Reasons: signs of a paper mill; compromised peer review; unreliable results or conclusions.

# Hybrid Optimized GRU-ECNN Models for Gait Recognition with Wearable IOT Devices

**DOI:** 10.1155/2022/5422428

**Published:** 2022-05-13

**Authors:** K. M. Monica, R. Parvathi, A. Gayathri, Rajanikanth Aluvalu, K. Sangeetha, Chennareddy Vijay Simha Reddy

**Affiliations:** ^1^School of Computer Science and Engineering, Vellore Institute of Technology, Chennai, Tamilnadu, India; ^2^Department of Computer Science and Engineering, Saveetha School of Engineering, Saveetha Institute of Medical and Technical Sciences, Chennai, India; ^3^Chaitanya Bharathi Institute of Technology, Hyderabad, Telangana, India; ^4^Department of Computer Science and Engineering, Kebri Dehar University, Kebri Dehar, Ethiopia; ^5^Department of Computer Science, Middlesex University, London, UK

## Abstract

With the advent of the Internet of Things (IoT), human-assistive technologies in healthcare services have reached the peak of their application in terms of diagnosis and treatment process. These devices must be aware of human movements to provide better aid in clinical applications as well as the user's daily activities. In this context, real-time gait analysis remains to be key catalyst for developing intelligent assistive devices. In addition to machine and deep learning algorithms, gait recognition systems have significantly improved in terms of high accuracy recognition. However, most of the existing models are focused on improving gait recognition while ignoring the computational overhead that affects the accuracy of detection and even remains unsuitable for real-time implementation. In this research paper, we proposed a hybrid gated recurrent unit (GRU) based on BAT-inspired extreme convolutional networks (BAT-ECN) for the effective recognition of human activities using gait data. The gait data are collected by implanting the wearable Internet of Things (WIoT) devices invasively. Then, a novel GRU and ECN networks are employed to extract the spatio-temporal features which are then used for classification to realize gait recognition. Extensive and comprehensive experimentations have been carried out to evaluate the proposed model using real-time datasets and also other benchmarks such as whuGait and OU-ISIR datasets. To prove the excellence of the proposed learning model, we have compared the model's performance with the other existing hybrid models. Results demonstrate that the proposed model has outperformed the other learning models in terms of high gait classification and less computational overhead.

## 1. Introduction

In recent years, activity recognition (AR) has witnessed exponential growth in in different domains such as healthcare [1], home automation [2], and even criminal activity detection. These methods are adopted aiming both at improving the quality of living and allowing people to stay without any support from others [3]. In the health care system, these AR systems are burgeoning technology mainly designed to detect the patient's mobility in rehabilitation therapy and to monitor physical performance after undergoing treatment with great expectations of improving his/her living quality as much as possible.

However, activity data remain more complex, which paid the way for the open research to design the intelligent human activity recognition system. Initially, simple binary sensors are used to design the recognition system [4, 5]. More recently, the Internet of Things (IoT) has been used to collect and analyze human activities and gestures [6, 7]. These devices are used as wearable devices that can be continuously used indoors or outdoors while ensuring the privacy and security of the data.

Owing to their pervasiveness and embedded sensor diversity, wearable IoT devices have been commonly used to develop AR recognition systems [8–10]. In this development, wearable IoT devices have the capability to capture and process activities and behaviors that are termed as gait signals. Accelerometers and gyroscopes are considered to be the most frequently used sensors equipped in WIOT devices to capture and transmit the gait sequences that can be used for further monitoring. Therefore, these devices have allowed for the extraction of diverse gait information from the person's movement that can be used to recognize physical activities related to health care applications.

Hence, the WIOT devices are considered as most important data capturing unit in AR systems. The collected data are then used to build the effective recognition systems. Magnificent development in AR systems is done by using the conventional machine learning algorithms such as Decision Trees [11–13], the Hidden Markov models [14–16], and support vector machines (SVMs) [17–19] have been deployed to achieve the higher rate of recognition. Since these methods are trapped in lower-dimensional data space, handling the larger data require the more efficient learning models to achieve higher performance.

Recently, studies are migrating towards deep learning algorithms to handle the larger amounts of data in an effective manner. Deep learning algorithms such as convolutional neural networks (CNNs) [20, 21] and recurrent neural networks (RNNs) [22, 23] play an undisputed role for developing AR systems. Additionally, the hybrid deep learning methods [24–26] are also gaining the brighter light of research in designing AR systems, but these collected gait data need transformation to influence the deep learning algorithms to obtain better classification with reduced computational cost. Hence, the hybrid combination of algorithms is required mandatorily to perform the data transformation and achieve high performance with low complexity.

In this context, this paper proposes a new hybrid algorithm, which ensembles the CNN layers with gated recurrent units and BAT-inspired classification networks. The user-defined CNN is used to extract the spatial features, whereas GRU is used to extract the temporal features. These features are then fed to complexity-aware BAT-inspired classification networks to achieve a better classification of AR with low complexity overhead.

### 1.1. Contribution

1. This paper focuses on the development of novel testbeds based on wearable IoT devices for the effective collection of raw gait data.
2. This paper also proposes a methodology for restructuring the raw data suitable to train the deep learning algorithms for better performance.
3. This paper proposes a hybrid deep learning algorithm for effective feature extraction with less computational cost and a high gait recognition rate.
4. Finally, the paper presents the excellence of the proposed methodology by conducting experiments using other benchmark datasets and comparing the performance with other existing deep learning-based AR systems.

The rest of the paper is organized as follows: Section 2 presents the related works proposed by more than one authors. The data collection unit, data preprocessing, and the proposed hybrid model are presented in Section 3. The dataset descriptions, experimentations, results, findings, and analysis are presented in Section 4. Finally, the paper is concluded in Section 5 with future enhancements.

## 2. Related Works

Abdullah et al. adopted a neural network for diagnosing the human abnormalities using their walking styles, which are detected at lower limbs. These real-time samples are extracted through the Levenberg-Marquardt method, and their artifacts are removed using the Butterworth filters in order to train the neural network effectively. The gait data are observed from 5-subjects at distinct speeds 2.4, 3.2, and 5.4 kmph and in total 45 instances are utilized for evaluation [27]. Though the proposed NN achieved better accuracy for tested data, it is not suitable for dynamic movements, and the tested data range are very low.

On the HuGaDB dataset, Saleh et al. used the three supervised machine learning models for human activity recognition: random forest, Navie Bayes, and IB1 classifiers. This HuGaDB contains data on standing, sitting, running, and walking, which is monitored using accelerometers and gyroscopes. Random forest outperformed the other two learning models in terms of classification accuracy while requiring less setup time [28]. Moon et al. introduced a multimodel gait identification classifier based on the convolutional and recurrent neural networks combined with a support vector feature extractor [29].

Jiang and Yin used the Short-time Discrete Fourier Transform (STDFT) to create a time-frequency-spectral image from time-serial signals in [30]. After that, CNN is used to process the image in order to recognize basic daily movements such as walking and standing. Using a mix of time-frequency-spectral characteristics and CNNs, Laput and Harrison [31] built a fine-grained hand activity sensing system. They were able to classify 25 atomic hand activities performed by 12 participants with a 95.2 percent accuracy. The spectral properties can be employed not only for wearable sensor activity recognition but also for activity recognition without the usage of a device. For learning modality-specific temporal properties, Ha and Choi [32] proposed a new CNN structure with distinct 1D CNNs for different modalities. Other types of CNN variants are being studied as part of the development of CNNs for efficiently integrating temporal characteristics.

Shen et al. [33] used the gated CNN to recognize everyday activities from audio signals and found it to be more accurate than the naïve CNN. Long et al. used residual blocks to create a two-stream CNN structure that can handle several time scales. On three benchmark datasets, Guo et al. [34] developed an ensemble technique of numerous deep LSTM networks that outperformed individual networks. Aside from RNN structure variations, other researchers looked into distinct RNN cells. For example, instead of using LSTM cells, Yao et al. [35] built an RNN using gated recurrent units (GRUs) and used it to activity recognition. However, some research has found that different types of RNN cells do not perform significantly better than the traditional LSTM cell in terms of classification accuracy [36]. Wang et al. [37] used the CNN and an LSTM to create a classifier that could automatically extract difficult characteristics from sound data and recognize gestures. For different scales of local temporal feature extraction, Xu et al. [38] used the sophisticated Inception CNN structure, whereas GRUs were used for efficient global temporal representations.

To assess more complex temporal hierarchies, Yuta et al. [39] used a dual-stream ConvLSTM network, with one stream handling shorter time lengths and the other longer time lengths. Guo et al. [40] proposed that MLPs be used to generate a base classifier for each sensory modality, and that ensemble weights be assigned at the classifier level to incorporate all classifiers. The authors not only evaluated recognition accuracy while creating the basis classifiers but also stressed variety by inducing diversity metrics. As a result, the diversity of different modalities is retained, which is important for overcoming over-fitting difficulties and enhancing overall generalization capacity.

## 3. Proposed System

### 3.1. System Overview

The proposed framework has four main phases, namely: (i) Data collection unit; (ii) Data preprocessing and filtering; (iii) Spatial and Temporal feature extraction using the proposed architecture; (iv) Classification phase. The block diagram of the proposed framework is shown in Figure 1.

### 3.2. Materials and Methods

#### 3.2.1. Data Collection Unit

To collect the experimental data, 29 volunteers with body weights ranging from 25 kg to 64 kg were selected. The participants were all healthy without any neurological disorders and had no physical injuries to their legs or feet, which may have affect the walking gait phase detection. With the advancement of Internet of Things (IoT) devices, this work used six battery-powered IoT devices to collect the corresponding inertial information. Figure shows the placement of the six IoT devices on the participants. To collect the inertial data from the lower limbs, MICOTT boards are used as the main IoT devices, which consist of 8-BIT NODEMCU as the main CPU interfaced with the 10-BIT SPI (Serial Peripheral Interface) based MCP3008 analog channels and ESP8266 WIFI transceivers. ADXL435 three-axis accelerometers and BMG250 three-axis gyroscopes are interfaced with MICOTT boards to collect inertial information from both limbs of participants. Micropython programming was deployed in the board to collect data and transmit them to the cloud. The series of Li-On batteries with operating voltage of 3.3 V is used to power up the board and can be replaced as the batter drains its total power.

During the experimentation, all participants were required to walk normally on the treadmill at different speed ranging from 0.66 m/s to 1.3 m/s for at least 180 s. All the participants were requested to walk normally for 2 minutes at each speed. The experimental data were collected for every 3 minutes and the data collected were transmitted to the cloud for further processing. Besides, to evaluate the excellence of the proposed algorithm, we have used other public benchmark datasets such as the whuGait and OU-ISIR datasets, and details of datasets are discussed in Section 4.  Figure 2 presents the data collection procedure used in the proposed methodology.

#### 3.2.2. Data Preprocessing Process

The stored data sample in the cloud contain multiple features from the six IoT devices, and each data includes acceleration and angular velocity data in the *X*, *Y* and *Z* directions. The sequences of the data sample are denoted by the following equation:

(1) $$\begin{array}{c} y=\left\{s1,f2,s2,f1,s3,f3\right\}, \end{array}$$

where *y* is the total data sample, *s*1, *s*2, and *s*3 are accelerometer data, and *f*1, *f*2, and *f*3 are angular velocity data, which are stored in cloud. As mentioned in the above equation, combined data are stored in the cloud, which need the segmentation and extraction that can be used for the better classification. The data collected in the cloud are downloaded offline and data preprocessing steps are used for effective data separation and extraction. To achieve less computational complexity with high accuracy of segmentation, this paper uses the novel Pearson correlation sliding window technique [41], which combines the Pearson correlation coefficient [42] and Sliding Window techniques. The value of *P* plays an important role in the data extraction, in which different thresholds are used for effective data extraction over a period of time.  Figure 3 presents the preprocessed data after applying the proposed technique.

#### 3.2.3. Proposed the Hybrid Deep Learning Model

As the analysis of the walking ability of the individual models with the fused features, we find that the integration of the different learning models can lead to better gait signal recognition and classification with less complexity. Hence, we intend to design the hybrid ensemble of the deep and machine learning models to learn the combined spatiotemporal feature effectively, which tends to the way of high accuracy and less computational complexity. The complete architecture of the proposed hybrid model is shown in Figure 4.

#### 3.2.4. CNN-Based Spatial Feature Extraction

This paper uses the CNN layers are core spatial feature extractors, which can act as the input to the dense learning layers, which are based on the optimized extreme learning machines. First, we briefly explain the concept of CNN architectures, which act as the main spatial feature extractor. The convolutional neural network (CNN) is a biologically propelled advancement of the multilayer perceptron (MLP).

As shown in Figure 5, CNN by connecting various convolution layers and max-pooling tasks. Information is handled through these profound layers to deliver the element maps, which are at last changed into an element vector by going through an MLP. This is alluded to as a fully-connected layer (FC) that performs classification and detection. For an effective spatial feature extractor, this paper uses six-convolutional layers in which the preprocessed collected data are given as the inputs. The CNN layers used in this paper are presented in Table 1.

The ReLU function is used as activation function in the network. To reduce the risk of the gradient vanishing problem, we used the batch-normalization process right after the fourth and fifth convolutional layers. The convolutional feature maps for the input *x* are denoted by using the following equation:

(2) $$\begin{array}{c} F=f\left(x,\left\{W1,B1,\beta \left(\text{Relu}\right)\right\}\right), \end{array}$$

where *W*1 is weight matrix of the layers, *b*1 is networks' bias weights, and *β*(Relu) is ReLU activation function. We train the network by initializing the weights randomly with a learning rate of 0.01 and momentum of 0.9.

#### 3.2.5. GRU-Based Temporal Feature Extraction

The most important structure used for the temporal feature extraction is the GRU module, which receives the data collected from the IoT-cloud systems.  Figure 6 shows the structure of the GRU network used in the paper.

The GRU network consists of two gates and is considered faster than the LSTM and RNN models [43]. Where *x*_*t*_ is the input feature at the current state, *y*_*t*_ is the output state, *h*_*t*_ is the output of the module at the current instant, *Z*_*t*_ and *r*_*t*_ are update and reset gates, *W*(*t*) is weights, and *B*(*t*) is bias weights at current instant. The mathematical expression for extracting the feature maps is given in the following equation:

(3) $$\begin{array}{c} P=\text{GRU}\left(\sum_{t=1}^{n}\left[x_{t,}h_{t,}z_{t,}r_{t}\left(W\left(t\right),B\left(t\right),\eta \left(\tan\;nh\right)\right)\right]\right). \end{array}$$

#### 3.2.6. Classification Layers

Next, we further propose an optimized single feed forward network, which uses the principle of extreme learning machine to train the spatio-temporal features obtained from the previous layers. In order to have less computational complexity, this research work uses the extreme learning network with auto-tuning property whose optimization is done by the BAT-inspired principles. The detailed description of the proposed classification layer is given as follows:

(1) ELM Decision and Classification layer: ELM is a kind of neural network that utilizes single hidden layers and works on the principle of auto-tuning property. ELM exhibits better performance, high speed, and less computational overhead when compared with the other learning models such as support vector machines (SVM), bayesian classifier (BC), K-nearest neighborhood (KNN), and even Random Forest (RF).

This kind of neural network utilizes the single hidden layers, in which the hidden layers do not require the tuning mandatorily. Compared with the other learning algorithms such as support vector machines (SVM) and Random Forest (RF), ELM exhibits better performance, high speed, and less computational overhead. ELM uses the kernel function to yield good accuracy for better performance. The major advantages of the ELM are minimal training error and better approximation. Since ELM uses auto-tuning of the weight biases and nonzero activation functions. The detailed working mechanism of the ELM is discussed in [44]. The input features maps of the ELM are denoted by the following equation:

(4) $$\begin{array}{c} X=F\left(F,P\right), \end{array}$$

where *X* is the fused spatio-temporal features obtained from the CNN and GRU layers, *F* is the CNN's spatial feature and *P* is the GRU temporal feature.

The output ELM function is denoted by the following equation:

(5) $$\begin{array}{c} Y\left(n\right)=X\left(n\right)\beta =X\left(n\right)X^{T}{\left(\frac{1}{C}XX^{T}\right)}^{-1}O. \end{array}$$

The overall training of ELM is given by the following equation:

(6) $$\begin{array}{c} S=\alpha \left(\overset{N}{\underset{n=1}{\sum }}\left(Y\left(n\right),B\left(n\right),W\left(n\right)\right)\right), \end{array}$$

where *X*(*n*) is input fused feature maps, *β* is temporal matrix, which is solved by the Moore−Penrose generalized inverse theorem, denoted by *X*^*T*^, *C* is constant, and *B* and *W* are weights and bias factors of the network with the sigmoidal activation function. The proposed network is trained with these features using the sigmoidal activation function. To resolve the computational problems, this paper adds the BAT-inspired optimizers to tune the hyper-parameters of the proposed ELM classifiers. The working mechanism of the BAT-inspired ELM is discussed as follows.

(2) BAT Inspired ELM Layers: this section describes the working mechanism of the BAT algorithm over ELM layers to provide better classification.

(3) Bat Algorithm- an Overview: the standard mega- bat calculation depended on the echolocation or bio-sonar attributes of microbats. In light of the echo cancelation calculations, Yang [45] (2010) built up the bat calculation with the accompanying three glorified guidelines:

1. All bats use echolocation to detect separation, and they likewise “know” the distinction between sustenance/prey and foundation obstructions in some mystical manner.
2. Bats look for prey by flying at a random velocity *v*_*i*_ at position *x_i_* with a fixed frequency fmin, changing wavelength λ, and loudness A0. They can consequently modify the wavelength (or recurrence) of their transmitted pulse and alter the rate of pulse emission *r* 2 [0, 1], based on the nearness of their objective.
3. In spite of the fact that the loudness can fluctuate from numerous points of view, we expect that the loudness shifts from an extensive (positive) *A*0 to a minimum constant value *A*min.

Each bat Motion is associated with the velocity *v*_*it*_ and initial distance *x*_*it*_ with the “*n*” number of iterations in a dimensional space or search space. Among all the bats, the best bat has to be chosen depends on the three rules, which are stated above. The updated velocity vit and initial distance *x*_*it*_ using the three rules are given below in the following equation:

(7) $$\begin{array}{c} f_{i}=f\min\pm \left(f\max-f\min\right)\beta ,\\ x_{it}=x_{it}-1+v_{it}, \end{array}$$

where *β* € (0,1) fmin is the minimum frequency = 0 and *f*max is the maximum frequency, which initially depends on the problem statement. Each bat is initially allocated for the frequency between the *f*min and *f*max. Consequently, bat calculations can be considered as a frequency tuning calculation to give a reasonable blend of investigation and exploitation. The emission rates and loudness basically give mechanism to programmed control and auto-zooming into the district with promising solutions.

To get a better solution, it is fundamental for the variety of the loudness and the pulse emission. Since the loudness normally diminishes once a bat has discovered its prey, while the rate of pulse emission expands, the loudness can be picked as any estimation of accommodation, between *A*min and *A*max, accepting *A*min = 0 implies that a bat has quite recently discovered the prey and briefly quit transmitting any stable.

#### 3.2.7. Advantages of Bat Algorithms

The major advantages of BAT algorithms are as follows:

1. High Efficiency than PSO, GA, and other heuristic algorithms [46]
2. Faster and more versatile search space than SGD [47]

Motivated by the advantages of the BAT algorithm, we proposed the new hybrid integration of the BAT algorithm and the ELM training network for better gait classification.

#### 3.2.8. BAT-Inspired ELM Layers

As discussed in Section 3.2.4, the simple bat algorithms are used to optimize the weights of ELM networks. In this case, bat's prey searching mechanism is used as the main term to optimize the weights and hidden layers of ELM. Initially, these hyper parameters are selected randomly and passed to the ELM training network. The fitness function of the proposed network is given by equation (9). For each iteration, hyper parameters are calculated by using equations (7) and (8). The iteration stops when the fitness function matches equation (9).

(8) $$\begin{array}{c} \text{Fitness Function}=\text{Max}\left(\text{Accuracy},\text{Precison},\text{REcall},\text{Specificty}\&\text{F}1-\text{Score}\right). \end{array}$$

Once the inputs weights are optimized by the BAT algorithm, the proposed classification layer classifies the gait activities with high speed and less computation. The working mechanism of the proposed classification layers is presented in Algorithm 1. The training network uses 30 epochs, batch size of 40 with 150 hidden layers and 0.001 learning rate.

## 4. Section -IV

### 4.1. Experimentation and Evaluation Metrics

Table 2 presents the experimental parameters used for training the proposed network. Furthermore, we have calculated the performance metrics such as accuracy, precision, recall, specificity, and F1-score using different datasets. Additionally, we have calculated the AUC (Area under ROC) and confusion matrix to prove the superiority of the proposed model. The mathematical expression used for calculating the performance metrics is presented in Table 3. Higher scores of the metrics indicate better performances. To solve the network's overfitting problem and improve the generalization problem, the early stopping method [48] is used in the paper. This method can be used to end the proposed network training when the validation performance shows no improvement for N consecutive times. The complete model was developed using open source TensorFlow version 2.1.0 with Keras as backend and implemented on a PC workstation with Intel Xeon CPU, NVIDIA Titan GPU, 16 GB RAM, and 3.5 GH_Z_ operating frequency.

### 4.2. Performance Evaluation of the Proposed Model Using the Different Datasets

In this part, we conducted experiments using real-time and benchmark datasets. We have calculated ROC and confusion matrix of the proposed network model using different datasets.

Figure 7 shows the ROC curves of the proposed model using different gait datasets. It is obvious that the proposed model has shown the 0.9880 AUC for raw data collected, 0.980 AUC for whuGait, and 0.9780 AUC for OU-ISIR datasets. The proposed network has shown constant performance for real-time datasets and public datasets also.  Figure 8-shows the confusion matrix of the proposed model using different dataset.  Figure 8 shows the confusion matrix of the proposed model under datasets. It is evident that from Figure 7, the proposed model maintains the uniform performance even with different datasets. The performance metrics of the proposed algorithm with the different datasets have been depicted in Table 4. From Table 4, it is found that the proposed network has exhibited higher performance using real-time datasets and whuGait datasets. It is also found that the proposed model has shown slight edge of peak performance when handling the OU-ISIR datasets.

### 4.3. Comparative Analysis of the Proposed Model with the Other Existing Models

To prove the superiority of the algorithm, performance of the proposed model is calculated and evaluated against the existing the hybrid deep learning algorithms such as TL-LSTM [49], 2D-CNN-LSTM [50], DCLSTM [51], Q-BTDNN [52], ATTENTION + CNN [53], CNN + GRU [54], and CNN + SVM [55].

Figures 9–14 show the performance of the different hybrid learning models using the IoT-based real-time datasets. It is found that the proposed hybrid model and CNN + GRU have exhibited the same performance in AR detection systems. But still, the proposed model has shown little edge over the CNN + GRU learning model and outperforms the other learning models in the detection of gaits. Figures show the comparative analysis of the different learning models using whuGait datasets. The proposed model has shown greater performance than the other existing learning models. The performance of the different learning models using OU-ISIR datasets are shown in Figures 9–14. From Figures 9–14, it is clear that the inclusion of the BAT-inspired ELM models along with spatio-temporal feature extraction has shown its excellence over the other learning models. From the above experiments, it is clear that the proposed model has shown the better AR rate even with multiple datasets.

### 4.4. Computational Complexity

The computational complexity of the proposed technique is represented by big-o-notations. The different CNN algorithms used for evaluation and complexity analysis are presented in Table 5. The mathematical expressions for calculating the computational complexity using Big-O-Notation are given by the following equation:

(9) $$\begin{array}{c} \text{Time Complexity }=\text{ O}\left(\text{Convolutaional layers}*\text{Pooling Layers}*\text{Training Networks}\right). \end{array}$$

From Table 5, it is found that BAT optimized classification layer has produced less computational complexity, which is even 10% lesser than the other existing algorithms.

## 5. Section -V

### 5.1. Conclusion and Future Scope

In this paper, a novel GRU fused CNN feature extractor with the BAT-inspired classification layer is formed for better recognition of human gaits that can be used for health care applications. The real-time datasets were collected using the wearable IoT(W-IoT) devices and stored in the cloud for further monitoring and processing. For an efficient classification, these data were restructured using the Pearson correlated sliding windowing method. Then, these restructured data are fed into the two layers of the deep learning model one is user-defined CNN, which is used to extract the spatial features and the other is GRU, which is used to extract the temporal features. Finally, these spatio-temporal features are then feed into the proposed BAT-inspired optimized classifiers to have better gait recognition. The extensive experimentation is carried out using the real-time datasets along with the public datasets such as whuGait and OU-ISIR benchmarks. Results demonstrated the proposed model has shown better recognition rate and less computational cost than the other existing hybrid learning models.

For future work, we would further implement the proposed gait recognition system over the limited hardware resource even on a smartphone. Besides, performance metrics, other parameters such as energy consumption, resource constraint parameters, and computing capability also to be considered for better implementation in real-world scenarios. Furthermore, our gait recognition model can extend its application toward the human behaviors prediction, which can play a vital role in psychology and crime investigation domains.

## Figures and Tables

**Figure 1:** Block diagram for the proposed methodology.

**Figure 2:** Data collection system used in the proposed methodology.

**Figure 3:** Data preprocessing after applying the proposed technique of data separation.

**Figure 4:** Proposed Architecture for the Hybrid Feature Extraction and Classification layer.

**Figure 5:** Schematic representation of convolutional neural networks.

**Figure 6:** GRU network for Temporal Feature Extractor.

**Figure 7:** ROC curves of the proposed methodology. (a) Real time Datasets; (b) Dataset-1(whuGait); (c) Dataset-2; (d) Dataset-3; (e) Dataset-4; (f) OU-ISIR datasets.

**Figure 8:** Confusion matrix for the Proposed Hybrid Model. (a) Real time Datasets; (b) Dataset-1(whuGait); (c) Dataset-2; (d) Dataset-3; (e) Dataset-4; (f) OU-ISIR datasets.

**Figure 9:** Performance analysis of the different hybrid models using real-time datasets.

**Figure 10:** Performance analysis of the different hybrid models using WhuGait Dataset-1.

**Figure 11:** Performance analysis of the different hybrid models using WhuGait Dataset-2.

**Figure 12:** Performance analysis of the different hybrid models using WhuGait Dataset-3.

**Figure 13:** Performance analysis of the different hybrid models using WhuGait Dataset-4.

**Figure 14:** Performance analysis of the different hybrid models using OU-ISIR datasets.

**Algorithm 1:** Pseudo Code for the Proposed Optimized ELM layers.

**Table 1:** Parameters of CNN spatial feature extraction.

Sl. No	No of convolutional layers	Stride length	No of layers
1	Conv(2d) -Layer-1	2	3 × 3
2	Max-pooling layers-1		2 × 2
3	Conv(2d) -Layer-2	2	3 × 3
4	Max-pooling layers-2		2 × 2
5	Conv(2d) -Layer-3	2	2 × 2
6	Max-pooling layers-3		1 × 1
7	Conv(2d) -Layer-4	2	2 × 2
8	Max-pooling layers-4		1 × 1
9	Conv(2d) -Layer-5	2	2 × 2
10	Max-pooling layers-5		1 × 1
11	Conv(2d) -Layer-6	2	1 × 1
12	Max-pooling layers-6	1 × 1	

**Table 2:** Training Parameters used for the Proposed Hybrid Model.

Sl. no	Detailed parameters	Specifications
01	No of Epochs	200
02	Batch Size	100
03	Learning Rate	0.0001
04	Training data	70
05	Testing data	30

**Table 3:** Mathematical expressions for the performance metrics' calculation.

Sl. no	Performance metrics	Mathematical expression
01	Accuracy	(TP+TN)/(TP+TN+FP+FN)
02	Recall	TP/(TP+FN) × 100
03	Specificity	TN/(TN+FP)
04	Precision	TN/(TP+FP)
05	F1-Score	2.((Precison*∗*Recall)/(Precision+Recall))

TP is True Positive Values, TN is True Negative Values, FP is False Positive and FN is False negative values.

**Table 4:** Performance metrics of the proposed model using different datasets.

Datasets	Performance metrics				
	Accuracy	Precision	Recall	Specificity	F1-score
Real-time Datasets	0.989	0.987	0.986	0.989	0.9902
Datasets-1	0.9889	0.985	0.984	0.978	0.983
Dataset-2	0.9890	0.9856	0.989	0.9902	0.989
Dataset-3	0.9890	0.9879	0.990	0.9901	0.992
Dataset-4	0.9891	0.9890	0.990	0.99	0.988
OU-ISIR datasets	0.990	0.989	0.982	0.992	0.990

**Table 5:** Computational complexity analysis between the hybrid and proposed model.

Algorithm Details	No. of layers required	Big-O-Notations

CNN (without Optimization)	No. of Convolutional layers = 6 No. of Polling layers = 06 No. of training layers = *k*	O (n6, n6, nk)
2DCNN-LSTM	No. of Convolutional layers = 05 No. of Polling layers = 05 No. of training layers = *k* + 3	O (n5, n5, nk + 3)
CNN-SVM	No. of Convolutional layers = 06 No. of Polling layers = 06 No. of training layers = *k* + 5	O (n6, n6, nk + 5)
CNN + GRU	No. of Convolutional layers = 06 No. of Polling layers = 06 No. of training layers = *k* + 6	O (n6, n6, nk + 6)
Attention CNN	No. of Convolutional layers = 06 No. of Polling layers = 06 No. of training layers = *k* + 10	O (n6, n6, nk + 10)
Proposed architecture	No. of Convolutional layers = 06 No. of Polling layers = 06 No. of training layers = k − 5	O (n5, n5, nk − 5)

^*∗*^ *k* = Maximum Number of required Training Layers.

## Data Availability

The data used to support the findings of this study are available from the corresponding author upon request (Sangeethak@kdu.edu.et).
